This article has been retracted.

# Occupational Therapy Practice Based on New-Generation Information Technology for Employee Emotion Analysis and Management

**DOI:** 10.1155/2022/3536911

**Published:** 2022-07-26

**Authors:** Yueyuan Cheng

**Affiliations:** Department of Foreign Languages, Zunyi Medical University (Zhuhai Campus), Zhuhai City 519000, China

## Abstract

This work intends to combine neural network technology with occupational therapy to fully acquire employees' emotional information by constructing an effective emotion recognition network. Firstly, the psychological state of employees is discussed from three aspects of leadership narcissism, organizational identification, and the emotional contagion effect, and the corresponding model is implemented. Secondly, based on the convolutional neural network technology, the facial feature recognition and the body feature recognition are combined, and the employees' emotions can be accurately identified by establishing a multilearning emotion recognition network. Finally, a questionnaire survey is carried out on the employees of enterprises in the coastal areas of Zhejiang. Descriptive statistical analysis, reliability and validity analysis, correlation analysis, regression analysis, mediation effect tests, and other methods are used to analyze the questionnaire data. The results reveal that leadership narcissistic organizational identification plays a mediating role in the process of employees' emotional contagion perception affecting employees' psychology. Compared with younger employees, older employees have better psychological quality and mental health. There are also significant differences in emotion and work enthusiasm among employees with different educational backgrounds and positions. Employees' perception of emotional contagion to pretending expressions, indifferent expressions, contempt expressions, and sincere expressions has an obvious positive impact on the psychological impact of other employees. The classification accuracy and regression error rate of the constructed multilearning emotion recognition network are 28.5% and 9.8%, respectively, which can accurately identify the emotional performance of employees. This work helps enterprises better understand the mental health of their employees.

## 1. Introduction

With the increasing development of the Internet, enterprises worldwide are experiencing great changes, transformation, and personalized development and need to be adjusted timely to adapt to the external environment that may change at any time [1]. This has a higher requirement for the managers of enterprises. The managers have to show the correct development direction for enterprises and employees when great changes take place. And they should fully believe in their employees and provide necessary resources to encourage employees to develop their innovation skills, ultimately increasing the profits of the enterprise and maintaining its advantages in competitions [2, 3]. And how to develop employees' innovation and arouse their work enthusiastic is an issue that needs to be studied. Some research teams around the world have researched how leaders drive employees' work passion to promote their innovation. In the research, many scholars pointed out that more attention should be paid to the mental health of employees in the process of developing their creativity [4]. Daud and Alfisah studied the decision-making ability and creativity of employees in a chemical fertilizer company in Indonesia and explored the role of psychological barriers in employees' innovation performance. A total of 200 questionnaires are distributed, and the data are collected by structural equation modeling (SEM). The results show that psychological barriers can reduce employees' performance and affect their decision-making ability, innovation performance, and creativity, thereby affecting their innovation performance [5].

Emotional contagion effect is also an important factor affecting employees' psychology. When employees' recognition of the enterprise is declined or even questioned, some leaders should use narcissistic methods to motivate their employees and guide them to find the direction of enterprise development [6, 7]. Wu and Wu studied the relationship between positive and negative emotional contagion and employees' innovation and the mediating effect of job engagement and employees' behavior. And the results show that job engagement plays a mediating role in the positive impact of employees' positive emotions on innovation behavior; employees' negative emotions play a mediating role in the supervisor's negative emotions and the influence of employees' behavior and innovation, but the role that they play is not significant [8]. However, few enterprises are willing to pay attention to employees' mental states, resulting in low efficiency. Also, some studied the impact of different types of leadership on employee management, and the results show that employees urgently need recognition from their leaders in the complex competitive environment. Conzelmann found that leaders could establish positive relationships with employees by recognition and rewards. This can help to retain employees who are essential to organizational development and improve employees' satisfaction, performance, and productivity [9]. In conclusion, most studies in this area have focused on the role of employee mental state in enterprise development and what can be done to improve employees' mental state. Previous studies have carried out a lot of research on employees' psychological barriers. The advantage is that the relationship between employee psychological barriers and employee innovation has been clarified. The disadvantage is that there are few studies on the impact of corporate executives on employees' psychology, and a large number of studies are mainly theoretical and less practical studies.

It is concluded that employees' mental states play an important role in improving their performance and enterprise development. Encouragement, rewards, and a good working environment can improve employees' satisfaction. However, there is no systematic research on the influencing factors of employees' mental states and their enthusiasm for work. Mental states directly affect the employees' enthusiasm for work, thereby affecting employees' performance and enterprise development. Employees' enthusiasm for work plays a mediating role in the leadership narcissistic organizational identification affecting employees' psychology. Moreover, employees' emotions can directly reflect their mental states. The traditional emotion recognition method extracts facial features for emotion judgment, but it has great limitations. Therefore, in the second part, the questionnaire design and processing are firstly carried out, and the employee's work motivation is used as an intermediate variable. Gender, age, education level, and position are used as control variables that affect the employee's psychological state, so that the conclusion is more accurate and scientific. Secondly, through the establishment of a multilearning emotion recognition network, facial feature recognition and body feature recognition are combined to achieve accurate recognition of employee emotions. Finally, the third part is the data statistics and analysis. It helps enterprises to better understand the mental states of employees, so that managers can understand employees' emotions at work through emotion recognition. And relevant measures are taken to carry out employees' emotional management and improve employees' enthusiasm for work, ultimately maximizing the interests of enterprises.

## 2. Questionnaire Design and Data Processing

### 2.1. Variable Analysis

- Relationship between leader narcissistic organizational identification and the mental health of employees

All the mental health and behaviors reflected by employees in their work are determined by the economic and emotional resources obtained by employees from the enterprise [10]. That is, the relationship between the employee and the enterprise is based on the principle of reciprocity. When the enterprise cares for employee's benefits and provides training opportunities for employees, employees may conduct different intrarole and extrarole behaviors for the enterprise, such as improving their performance and safeguarding the interests of the enterprise. Social learning theory believes that people often intentionally or unintentionally imitate the behavior of the model around them, and take the model's behavior as a goal to make corresponding adjustments and changes to their behavior [11–14].

(B) Relationship between employees' emotional contagion perception and leader narcissistic organizational identification

Social identification theory argues that employees would compare their own enterprises with others' to form a basic cognition to their enterprises, which may change employees' mental health sometimes. A good social reputation and image can bring positive cognition to employees and have a positive effect on employees' mental health [15, 16]. If an enterprise takes the social responsibility for external stakeholders, this will make their employees feel proud to be members of the enterprise and identify with corporate culture, and being loyal to the enterprise, thereby enhancing the social influence of the enterprise [17].

Social identification theory also points out that the decisions made by enterprises affect the employees' attitudes towards enterprises, and organizational identification has a positive impact on employees' behaviors [18, 19]. Social responsibility makes employees believe that their enterprises are responsible and enhances employees' recognition of the enterprise. Good organizational identification can stimulate employees to have high-quality organizational behavior. This shows that employees will feel proud, attached, and belonging and identify with corporate culture and reward the enterprise by a series of organizational citizenship behavior, if the enterprise takes corporate social responsibility to external stakeholders or fulfills the corporate social responsibility to internal employees.

(C) Relationship between narcissistic organizational identification and leadership effectiveness

Studies show that narcissism is positively correlated with leadership effectiveness. For example, a longitudinal study of military cadets shows that narcissism is positively correlated with self-leadership development and performance. Kotera et al. found that the change of leadership styles reported by superiors was positively correlated with narcissism [20]. They took the President of the United States as the research sample and found that narcissism of the President of the United States is positively correlated with personal charm and performance, and narcissism personality traits were more common in the group of the President. Typically, such leaders are also President Roosevelt of World War II, President Nixon, and the new U.S. President Kawab. The research proves that narcissism plays a positive role in promoting the mental health of their employees. Since narcissistic leaders attach great importance to their images, subordinates usually feel that their superiors are very attractive. At the same time, narcissistic people often have a certain pursuit of power and become charismatic and authoritative leaders. Feinstein et al. believed that constructive narcissistic leadership would improve the perception of psychological empowerment. Some studies show that there is a negative relationship between narcissism and leadership. In the sample study of a group of CEOs of the American Professional Baseball Association, it is found that narcissism is negatively correlated with leadership because narcissists are less likely to promote the establishment of a fair exchange relationship [21].

(D) The mediating effect of organizational identification

The organizational identification is taken as the mediating variable to study the influence of social responsibility awareness on organizational citizenship behavior, and its role between the two is explored.

(E) Establishment of the model

The main content is the impact of corporate social responsibility awareness on organizational citizenship behavior and the influence mechanism from multiple perspectives. The theoretical research model is shown in Figure 1.

Figure 1 shows that the selection of organizational identification variables in the model plays a mediating and moderating role in the whole model. The full or partial mediating role of organizational identification between corporate social responsibility awareness and organizational citizenship behavior is verified.

### 2.2. Questionnaire Design

- Scale selection

Mature scales developed by foreign scholars are used to measure organizational identification, employee emotional contagion, employee mental health, and employees' work enthusiasm. The good reliability and validity of these scales have been confirmed by many scholars in China and foreign countries. After the relevant literature is reviewed, it is found that the influencing factors, including gender, age, education, the nature of the enterprise, and posts, may affect the research variables. Therefore, the control variables are gender, age, education, and posts. This study mainly uses four scales to collect data [18, 22]. All measurement scales are scored by the Likert 5 scoring method, and 1–5 points correspond to the options from “total inconformity” to “total conformity,” respectively.

1. Employees' emotional contagion perception scale: the scale is developed by Turker in 2009 and includes 17 items, which can be divided into four dimensions: pretending expression, indifference expression, contempt expression, and sincere expression [23]. And it is widely used by a large number of relevant research teams and meets the needs of the definition and measurement of employees' emotional contagion perception. Cronbach's *α* of the scale is 0.87
2. Organizational identification scale: the organizational identification questionnaire, which is developed by Mael and Ashforth in 1992, is selected according to the needs of this study, and it has six items. Cronbach's *α* of the scale is 0.85
3. Employees' mental scale: the existing studies show that the scale developed by Williams and improved by Lee and Allen in 2002 is selected because of its rich structure, and it has 11 items [24]. And its reliability and validity are proved by many domestic and foreign scholars in empirical research. The scale is divided into two dimensions: “employees' mental health in profit-making enterprises” and “employee mental health in employee-benefiting enterprises.” The number of items in each dimension is 5 and 6, respectively. Cronbach's *α* of the scale is 0.89
4. Employee work enthusiasm scale: the workplace gossip scale developed by Brady et al. in 2017 is selected to evaluate employees' work enthusiasm, and it includes two dimensions of employees' positive and negative attitudes towards work [25] with four items in each. Cronbach's *α* of the subscale is 0.93

(B) Questionnaire design

The mature scale developed by foreign scholars is used to measure leadership narcissistic organizational identification, employees' emotional contagion, employees' mental health, and their work enthusiasm. All scales are analyzed by the Likert 5-level scoring method (1 = completely inconsistent, 2 = inconsistent, 3 = general, 4 = consistent, and 5 = fully consistent). The first part of the questionnaire is the basic personal information, which includes gender, age, education, the nature of the enterprise, and posts [26]. And the second part is the employee emotional contagion perception scale, the third is the leadership narcissistic organizational identification scale, the fourth is the employee psychological scale, and the fifth part is the employee work enthusiasm scale. In addition, the purpose of the survey is described in detail at the beginning of the questionnaireaccording to the principles of rigor and confidentiality.

(C) Sample selection and questionnaire distribution

The enterprises or institutions that belong to the following three types are selected as the research objects: communication enterprises, e-commerce enterprises, and Internet enterprises [27]. The questionnaires are mainly distributed in the coastal areas of Zhejiang to the intellectual personnel in the enterprises. A total of 300 questionnaires are distributed. After 32 invalid questionnaires are excluded, the number of valid questionnaires is 268, and the effective rate is close to 89%. All the questionnaires have been recovered, and the 32 invalid questionnaires refer to those with missing answers.

(D) Questionnaire data processing methods

SPSS 25.0 is used to test the data obtained from the questionnaire. The data analysis methods used are as follows:

1. Descriptive statistical analysis: SPSS 25.0 software is used for the preliminary descriptive statistical analysis of the survey data. The median, variance, and standard deviation of each demographic variable in the survey data are obtained [28]
2. Reliability and validity analysis: the reliability of the scale is analyzed by using the reliability measurement function button in SPSS 25.0 software, aiming at the consistency and reliability of the test variable data. The factor analysis method is used to measure the questionnaire, and validity analysis is conducted on the results. Validity analysis is to test whether the measurement results of the questionnaire can predict the accurate content and models [29]
3. Independent sample *T*-test and one-way ANOVA. Independent sample *T*-test is used to test the difference between the two groups. The independent variable is binary, and it is a continuous variable [30]
4. Correlation analysis: correlation analysis is mainly used to analyze the linear correlation between the variables. Pearson analysis in SPSS25.0 software is used to calculate the correlation coefficient *r* and the significance value, and these data are used to prove the correlation between each variable
5. Regression analysis: based on the above verification of the correlation between variables, a regression equation model is established to analyze the causal relationship between variables, that is, whether the change in the value of one variable causes the change in the value of another variable [31]
6. Mediation effect tests: combined with the mediating effect test method used by Wen Zhonglin, the variables in this questionnaire are tested

Questionnaires are used to know about the factors affecting the mental states and work enthusiasm of employees in enterprises in Zhejiang. On this basis, the corresponding strategies are proposed to implement employees' emotion management, hoping to improve employees' satisfaction with the enterprise through reasonable management methods and enhance their enthusiasm for work.

Based on the above content, the following assumptions are made:

1. Employees' emotional contagion perception and corporate customer's emotional contagion perception have a positive impact on employee psychology and employee emotional contagion perception of cooperative enterprises
2. Employee emotions have a positive and significant effect on the leadership narcissistic organizational identification, and employees' emotional contagion perception has a significant positive effect on other employees
3. Leadership narcissistic organizational identification has a significant positive influence on employees' mental health, and organizational identification has an obvious positive impact on employees' mental health in for-profit and employee-beneficial enterprises

### 2.3. Employees' Emotion Recognition

- Scene feature extraction network

The scene feature extraction network takes the whole image containing many people as the input to extract the global features of the scene. VGG16 is first used for pretraining on the database to speed up the training efficiency. The scene feature extraction network contains four dense feature modules, each of which reduces the number of channels for input feature mapping through two 1 × 1 convolution kernels.

(B) Body feature extraction network

The body feature extraction network takes the implicit facial expression, head position, and body posture information in the image as the input, and it is similar to the scene feature extraction network. The body feature extraction network is composed of five convolution layers and an end-to-end structure composed of a fully connected layer. The BN (batch normalization) layer, the pooling layer, and the ReLU layer are connected after each convolution layer to improve the nonlinearity of the network. The pooling layer can prevent the overfitting of the feature map, reduce the dimension of the feature map, and better retain the global information of the input feature map.

(C) Fusion decision network

The feature information output by the scene feature and body feature network is reconstructed and brought into the fusion decision network. The network performs convolution operation by a 1 × 1 convolution kernel and a 3 × 3 convolution kernel and splices all output results. Different convolution operations can obtain different information about the input image, and the feature mapping after parallel operation shows stronger feature representation ability [32]. Furthermore, six composite layers are used to establish direct connections between different layers, making full use of the feature mapping of each layer and combining the characteristics of each channel to alleviate the gradient disappearance problem. Also, the batch normalization layer and the ReLU function are used in each layer to further prevent the gradient disappearance and gradient explosion and increase the nonlinearity of the network. The final output includes two parts: multilabel emotion classification and continuous spatial emotion regression.

### 2.4. Research on Loss Function in Network Task

Since the multilabel emotion classification in the model is a classification task, the continuous spatial emotion regression is a regression task and the two tasks adopt different loss functions.

The global loss function *F* is the weighted sum of two different loss functions defined as

(1) $$\begin{array}{c} F=\lambda_{1}F_{\text{ML}}+\lambda_{2}F_{\text{G}}. \end{array}$$

*F*_ML_ and *F*_G_ are multilabel classification and continuous variable regression loss functions, respectively. *λ*_1_ and *λ*_2_ are different loss weights. Here, several different loss function combination schemes are tested, and they are introduced in detail below.

- Multilabel classification loss

Because of the label imbalance in multilabel sentiment classification, an improved *F*_L_ (focal loss) function is proposed. The focus loss function is one of the commonly used methods in dealing with sample imbalance in the field of target detection [33]. The mechanism of this function is to assign more weights to small samples or hard-to-class samples to improve the attention of these samples. In general, the focus loss function *F*_L_ is defined as follows:

(2) $$\begin{array}{c} F_{\text{L}}\left(\sigma_{\text{t}}\right)=-\alpha {\left(1-\sigma_{\text{t}}\right)}^{\gamma }\log_{n}\left(\sigma \text{t}\right), \end{array}$$

(3) $$\begin{array}{c} \sigma_{\text{t}}=\left\{\begin{array}{cc} \sigma , & \text{if}y=1,\\ 1-\sigma , & \text{else}. \end{array}\right. \end{array}$$

In equation (3), *γ* is the focus parameter amd *σ* and *γ* are the classification model output and the real label of the positive samples, respectively. The sentiment classification has the problems of sample imbalance and multilabel classification. Therefore, the improved focus loss function *F*_ML_ is defined as follows to improve the efficiency of the multi-label sentiment classification:

(4) $$\begin{array}{c} F_{\text{ML}}\left(y,\sigma \right)=-\overset{\text{Mc}}{\underset{i=1}{\sum }}\;\alpha {\left(1-\sigma_{i}\right)}^{\gamma }y_{i}\log_{n}\left(\sigma_{i}\right)+\left(1-\alpha \right)\sigma_{i}^{\gamma }\left(1-y_{i}\right)\log_{n}\left(1-\sigma_{i}\right). \end{array}$$

In equation (4), Mc is the number of categories (Mc = 26 in this study), *σ*_i_ and y_i_ are the classification model output and the *i*th true tag, respectively, and *α* and *γ* are the hyperparameters. *α* is used to set the recall rate or precision ratio, and *γ* is the focus parameter, which is the same as the traditional focus loss parameter. The main function of *γ* is to increase the weight of difficult classification samples and reduce the weight of easy classification samples to improve the overall sample balance.

In addition, the classification loss functions such as cross-entropy and Euclidean distance, and the regression losses such as Huber loss, mean square deviation loss, and average absolute error are compared and analyzed to explore the operation performance of the proposed loss function. The cross-entropy and Euclidean distance loss function *F*_C_ and *F*_E_ are defined as follows:

(5) $$\begin{array}{c} F_{\text{c}}\left(y,\sigma \right)=\overset{\text{Mc}}{\underset{i=1}{\sum }}y_{i}\log_{n}\left(\sigma_{i}\right)+\left(1-y_{i}\right)\log_{n}\left(1-\sigma_{i}\right),\\ F_{\text{E}}\left(y,\sigma \right)=\overset{\text{Mc}}{\underset{i=1}{\sum }}\;{\left(\sigma_{i}-y_{i}\right)}^{2}. \end{array}$$

(B) Continuous variable regression loss

Two different measurements are used to analyze the regression loss. Mean square error loss *F*_G_^*L*_2_^ and mean absolute error *F*_G_^*L*_1_^ are defined as follows:

(6) $$\begin{array}{c} F_{\text{G}}^{L_{1}}\left(y,\sigma \right)=\frac{1}{M_{G}}\overset{M_{G}}{\underset{i=1}{\sum }}\;\left|\sigma_{i}-y_{i}\right|, \end{array}$$

(7) $$\begin{array}{c} F_{\text{G}}^{L_{2}}\left(y,\sigma \right)=\frac{1}{M_{G}}\overset{M_{G}}{\underset{i=1}{\sum }}\;{\left(\sigma_{i}-y_{i}\right)}^{2}. \end{array}$$

In equations (6) and (7), *σ*_i_ and y_i_ are the same as the previous parameters. *M*_*G*_ is the dimension of continuous variables, and it is taken as 3.

The simulation compiler environment uses pytorch1.5.1+CUDA10.0 to build the network in python language. The simulation hardware environment is as follows: NVIDIA rtx2080ti 11 GB, Linux operating system.

## 3. Data Statistics and Analysis

### 3.1. Descriptive Statistical Analysis

Figure 2 below shows the descriptive statistical analysis.

From the data of the sample in Figure 2, men accounted for 56.3% and women accounted for 43.7%. Those aged 20 and below accounted for 0.7%, those aged 21-30 accounted for 57.8%, those aged 31-40 accounted for 8.7%, and those aged 51 and above accounted for 0.3%. In the education survey, the proportion of people with a bachelor's degree is the highest, over 70%, followed by a master's degree or above at 20.1%, a junior college degree at 9.0%, and a high school education or below at 0.4%. In this study, 78.7% of the employees are primary-level employees, followed by middle-level managers, accounting for 18.7%, and the proportion of senior managers is the least at 2.6%. It can be seen that most of the subjects were between the ages of 21 and 30, followed by subjects aged 31-40. Most of the main positions are grassroots workers. In general, the subjects of the study are young, highly educated knowledge-based employees. Among the subjects, general staff accounted for the largest proportion (78.7%). The higher the post, the less the subject, which conforms to the pyramid structure.

### 3.2. Analysis of the Reliability and Validity of the Scales

- Reliability analysis

The values of Cronbach's *α* of the scale and four variable scales (the organizational identification scale, the employees' emotional contagion scale, the employees' mental health scale, and the employees' work enthusiasm scale) are obtained. The statistical results are shown in Figure 3.

The standardized values of Cronbach's *α* of the four scales sre all greater than 0.8, indicating that the used scales has high reliability and passes the reliability test. The standardized values of Cronbach's *α* of the organizational identification scale, the employees' emotional contagion scale, the employees' mental health scale, and the employees' work enthusiasm scale are all around 0.9, illustrating scales have good reliability and stable measurement.

(B) Validity analysis

Figure 4 shows the validity analysis of each scale.

The above figure shows that the KMO (Kaiser-Meyer-Olkin) values of leader narcissistic organizational identification scale, employees' emotional contagion scale, employees' mental health scale, and employees' work enthusiasm scale are all above 0.7, indicating that these four scales are very suitable for structural validity analysis. The KMO values of each scale are greater than 0.7 or around 0.7, and the Bartlett spherical test results are significant (significant values are 0.000 < 0.01), indicating that the correlation between variables is strong and independent. This proves that the results of the questionnaire survey are suitable for structural validity analysis.  Figure 5 is the results of the fitting index test.

The above figure shows that the fitting indexes of the four-factor model are acceptable and effective, and the four variables have good validity and can be used to verify the subsequent hypothesis. This proves that the fitting indexes of the four scales mostly meet the requirements, and some indexes are very excellent, indicating that the fitting effect of data and model is good.

### 3.3. Analysis of Variance

- One-way analysis of variance of the employees' ages

Figure 6 shows the results of variance analysis of the employees' ages.

There are significant differences between the age groups of 21–30 and 41–50 in the perception of leader narcissistic organizational identification and the negative attitude of employees towards work. The perception of leader narcissistic organizational identification and the negative attitude towards work of employees aged from 21 to 30 are higher than those of the age group of 41–50. The reason may be that when employees are older, their experience and experience are richer. Older employees have a more serious and positive attitude towards the organization's social responsibility, and they are more willing to obtain leadership recognition through hard work and positive attitudes.

(B) One-way analysis of variance of employees' education

Figure 7 below shows the results of variance analysis of employees' education.

Figure 7 shows that the *F* values of employees with different educational backgrounds are maintained between 2 and 2.7, indicating that the educational background has a significant difference in employee emotions and work enthusiasm. Employees with a college degree have a significantly higher level of organizational identification than those with a master's degree or above. This may be because employees are more able to adjust their working states and moods through their perception of the organizational characteristics.

(C) One-way analysis of variance of the employees' posts

Figure 8 below shows the results of variance analysis of the employees' posts.

The results of the above figure show that posts have a great influence on employees' mental health and work enthusiasm. The organizational citizenship behavior of top managers is significantly less than that of the grassroots workers and middle-level managers. The possible reason is that top managers serve the enterprise for years and are ready to make more contributions to the organization. Therefore, their organizational citizenship behavior is less.

### 3.4. Correlation Analysis of Variables

The Pearson correlation analysis method is used to analyze the correlation between variables.  Table 1 below shows the statistical results of the correlation coefficients of the variables.

The above data show that the pretending expression, indifferent expression, contempt expression and sincere expression, leader narcissistic organizational identification, employees' mental health of profitable–making enterprises, employee-benefiting enterprises, and their dimensions are significantly correlated with employees' positive and negative attitudes towards work. Specifically, there is a significant positive correlation between the dimensions of employees' emotional contagion perception and those of leader narcissistic organizational identification and employees' mental health. There is a significant positive correlation between the dimensions of employees' positive attitudes towards work and those of employees' emotional contagion perception, organizational identification, and employees' mental health. There is a significant negative correlation between the dimensions of employees' negative attitudes towards work and those of leader narcissistic organizational identification and employees' mental health.

### 3.5. Regression Analysis of Variables

- The regression of employees' perception of emotional contagion to organizational citizenship behavior

Figure 9 below shows the statistics of the regression coefficient.

Figure 9 shows that the regression coefficients of each variable remain between 1 and 3, indicating that there is no multicollinearity among variables. And the satisfaction of employees remains between 13 and 18, which indirectly shows that employees' emotional contagion perception and its dimensions have a positive and significant impact on employees' psychology. Employees' emotional contagion perception and enterprise customers' emotional contagion perception have a positive effect on employees' psychology and employees' emotional contagion perception of cooperative enterprises.

(B) Regression analysis of corporate social responsibility perception on organizational identification

Figure 10 below shows the regression coefficient of employees' emotional contagion perception on leader narcissistic organizational identification.

According to the statistics of the above data, it is found that pretending expression, indifferent expression, despise expression, and sincere expression have a positive and significant effect on leader narcissistic organizational identification. And they have a positive and significant effect on the mental health of other employees, and the employees' emotional contagion perception has a significant positive effect on other employees.

(C) Regression analysis of leader narcissistic organizational identification on employees' mental health

Figure 11 below is the statistics of the regression coefficient of organizational identification on employees' mental health behavior in profit-making enterprises and employee-benefiting enterprises.

According to the statistical results of Figure 11, it is found that in the regression analysis of leader narcissistic organizational identification on employees' psychology, the significance is 0, which is smaller than 0.01, and the regression effect is obvious. Leader narcissistic organizational identification has a significant and positive impact on employees' mental health. Based on the above statistical analysis data, this regression equation has a good regression effect. This indicates that organizational identification has a significant and positive impact on employees' mental health in profit-making enterprises. Organizational identification has an obvious positive effect on employee mental health of profit-making and employee-benefiting enterprises.  Figure 12 below shows the results of the test of the mediating effect of leader narcissistic organizational identification.

Figure 12 shows that Model 1 and Model 2 take leader narcissistic organizational identification as dependent variables and Model 3, Model 4, and Model 5 take employees' psychology as the dependent variable. Model 1 and Model 2 only add the control variables set to test the mediating effect of leader narcissistic organizational identification by comparison. Three steps correspond to models 2, 4, and 5 in the table above. Based on Model 4, the intermediary variable of the organizational identification is introduced in Model 5, and the regression results of Model 4 and Model 5 are compared. The results show that after leader narcissism organizational identification is added, Δ*R*^2^ = 0.05 and *p* value is less than 0.01, indicating that the variance explained by the regression equation increases significantly, and the regression model used has a good fitting effect. The regression of the impact of employee emotional contagion perception on employees' psychology decreases significantly, from 0.61 to 0.44, and the regression coefficient of leader narcissism organizational identification is significant, with a value of 0.27.Therefore, leader narcissistic organizational identification plays a partial mediating role in the influence of employees' emotional contagion perception on employees' mental health.

### 3.6. Simulation and Analysis

This simulation compilation environment uses pytorch1.5.1+CUDA10.0 to build a network in python language. The simulated hardware environment is as follows: NVIDIA rtx2080ti 11 GB and Linux operating system.  Figure 13 shows the accuracy of employees' emotion analysis.

Figures 13(a) and (b) show that curve A shows the final loss training effect composed of the Euclidean distance classification loss and the average absolute error regression loss. It is found that the training of about 80 generations under this combination tends to be stable, and the average accuracy finally converges to 28.10%. Curve B shows the loss training effect composed of the Euclidean distance classification loss and the mean square deviation loss. In this combination, the training of about 80 generations tends to be stable, and the average accuracy eventually converges to 28.30%. Curve C shows the combined training effect of the improved focus loss and the average absolute error regression loss. In this combination, the training of about 20 generations tends to be stable, and the average accuracy eventually converges to 28.50%. Curve D shows the loss training effect composed of the improved focus loss and the mean square error loss. The training of about 110 generations in this combination tends to be stable, and the average accuracy eventually converges to 28.00%. Curve E shows the loss training effect composed of the cross-entropy loss and the mean square deviation loss. The training of about 120 generations in this combination tends to be stable, and the average accuracy eventually converges to 27.20%. Curve F shows that the loss training effect is composed of the cross-entropy loss and the average absolute error regression loss. The training of about 110 generations in this combination tends to be stable, and the average accuracy eventually converges to 27.40%.  Figure 13(c) shows the comparison of the average error rate of continuous regression under different loss combinations. Similarly, the average error rate in the A curve converges to 0.12, converges to 0.12 in the B curve, converges to 0.10 in the C curve, converges to 0.12 in the D curve, converges to 0.13 in the E curve, and converges to 0.12 in F curve. The comprehensive analysis of the improved focus loss and the average absolute error regression combination loss shows better training performance. Under this combination, the training speed is fast and the average accuracy of the classification and the average error rate of regression are 28.50% and 9.80%, respectively, which can more accurately identify the emotions of employees in the enterprise.

### 3.7. Strategies for Employees' Emotion Management

1. Guiding employees to establish correct emotional management concepts

Concepts play important roles in guiding people's behaviors. Therefore, in the process of enterprise management, it is necessary to actively guide employees and managers to attach importance to emotional management, so that they can realize that positive emotions have great significance to the completion of their tasks. Emotional management should be carried out throughout the entire process of employees' management. In the talent recruitment and selection, enterprises should hire the the employees who are good at emotional control. And then, timely attention should be given to the emotional trends of employees and corresponding adjustments should be made actively, so that a reasonable and effective system to maintain the positive emotions of employees is created.

(2) Employing various incentives

Effective incentives can help to maintain the positive emotions of employees. Therefore, care and help should be given to their work, life, and emotions according to the characteristics and needs of different employees. Reasonable and fair distribution systems should be established to improve employees' satisfaction, and an effective performance evaluation system is built to evaluate emplyees' performance reasonably and mobilize employees' enthusiasm for work, so that the positive emotions of employees at work are stimulated.

(3) Actively eliminating employees' negative emotions

Managers must take measures to relieve employees' pressure, so that they can find ways to release their negative emotions, provide employees with cultural and recreational activities, and maintain the positively mental state of employees at work. Standardized and orderly communication channels between employees and managers at all levels are established, and employees' opinions and suggestions can be timely reponded timely, eliminating employees' negative emotions.

(4) Enriching corporate culture and incorporating emotional management into corporate culture construction

Compared with the emotions of employees, managers of enterprises should undoubtedly pay more attention to the shaping of organizational emotions and corporate emotions. And there is a very close relationship between corporate emotions and employees' concepts in corporate culture. The relationship is the external manifestation of corporate values and employees'mental states. Therefore, managers at all levels, especially senior managers, should pay attention to the cultivation of corporate sentiment in cultural construction. In the construction of organizational culture, great importance should be attached to organizational emotions and other work.

## 4. Discussion

The characteristics of the research object are 21-30 years old, the education is mainly undergraduate, and the position is the grassroots employee. This is basically consistent with the current state of the labor force in China. As employees are older and have richer experiences, older employees have a more serious and positive attitude towards the organization's social responsibility, and they are more willing to gain recognition from leaders through their hard work and positive attitude. In the research on employee social responsibility and age, Nyuur et al. also believed that employee age was proportional to social responsibility [34]. A more specific analysis is carried out, and it is concluded that there is no specific correlation between employees' education and organizational identification. In the research on employee emotions, there is a significant positive correlation among the employee's emotional contagion perception dimension, the leadership narcissistic organizational identification dimension and the employee's mental health dimension. There is a distinct positive correlation among employees' positive attitude towards work and employees' emotional contagion perception, organizational identity and employees' mental health. The emotional contagion perception of employees and the emotional contagion perception of corporate customers have a positive impact on the employees' psychology and employees' emotional contagion perception of cooperative enterprises. Leadership narcissistic organizational identification has a significant positive impact on employees' mental health, and it plays a partial mediating role in the impact of employees' emotional contagion perception on employees' mental health. So far, the assumptions are all established. In the research on employee emotions and leadership narcissistic organizational identification, Surliuga believed that employee emotions were affected by leadership narcissistic organizational identification, but did not analyze the specific impact [35]. On this basis, it carried out a specific analysis of employees' mental health and positive attitudes, enterprise customers' emotional contagion, and so on.

## 5. Conclusion

The influencing factors of employees' psychological state and work enthusiasm under leadership narcissistic organizational identification are explored. Taking the employee's enthusiasm as an intermediate variable, and taking gender, age, education level and position as the control variables that affect the employee's mental state and work enthusiasm, the relevant model is realized. The results manifest that leadership narcissistic organizational identification plays a partial mediating role in the perception of employees' emotional contagion. The emotional contagion of employees' pretending, indifferent, contemptuous, and sincere expressions has a significant positive influence on the psychological impact of other employees. Employees' emotional management can guide employees to establish correct emotional management concepts through the use of various incentives, relieve employees' pressure, and actively eliminate employees' negative emotions, enrich the connotation of enterprise culture, and incorporate emotional management into the construction of enterprise culture. The classification accuracy and the regression error rate of the constructed multilearning emotion recognition network are 28.5% and 9.8%, respectively, which can accurately identify the emotional performance of employees. But there are still some limitations: the research object is in the coastal area of Zhejiang, which belongs to the economically developed area of China. Therefore, the results cannot bring practical reference to enterprises across the country. In-depth analysis should be conducted from the perspective of senior managers, rather than one-sided data analysis from the perspective of researchers. This research helps enterprises better understand the psychological state of employees, and enterprise managers can understand employees' emotions at work through emotion recognition and take relevant measures to manage employees' emotions, improve employees' work enthusiasm, and ultimately maximize the interests of the enterprise.

## Figures and Tables

**Figure 1:** The theoretical research model.

**Figure 2:** Descriptive statistical analysis ((a) gender, (b) age, (c) education, and (d) posts).

**Figure 3:** Statistical analysis of Cronbach's *α* (A: organizational identification scale; B: employees' emotional contagion scale; C: employees' mental health scale; and D: employees' work enthusiasm scale).

**Figure 4:** Validity analysis (a) validity analysis of organizational identification scale and employees' emotional contagion scale. (b) Validity analysis of employees' mental health scale and employees' work enthusiasm scale. A: approximate chi-square. B: degree of freedom. C: significance. D: the statistical test of the four scales).

**Figure 5:** Fitting detection (A: *λ*2); B: *Df*; C: goodness of fitting index; D: comparison of the fitting index; E: fitting index model; and F: root mean square of the approximation error).

**Figure 6:** The results of variance analysis of the employees' ages (A: less than 20 years old; B: 21-30 years old; C: 31-40 years old; D: 41-50 years old; and E: over 50 years old).

**Figure 7:** Analysis of variance of the employees' education (A: high school education and above; B: associate degree; C: bachelor's degree; and D: master's degree and above).

**Figure 8:** The results of variance analysis of the employees' posts (A: grassroots workers; B: middle-level managers; and C: top managers).

**Figure 9:** Result statistics of the regression coefficient of each variable ((a) pretending expression, (b) indifferent expression, (c) contempt expression, and (d) sincere expression. A: *B* value in nonstandardized coefficient; B: standard error in nonstandardized coefficients; C: standardization coefficient; D: *t* value; and E: Sig.).

**Figure 10:** Statistics of the regression coefficient of the employees' emotional contagion to leader narcissistic organizational identification ((a) pretending expression, (b) indifferent expression, (c) contempt expression, and (d) sincere expression. A: *B* value in nonstandardized coefficient; B: standard error in nonstandardized coefficients; C: standardization coefficient; D: *t* value; and E: Sig.).

**Figure 11:** Regression analysis of leader narcissistic organizational identification on employees' mental health ((a) employees' mental health in profit-making enterprises and (b) employees' mental health in employee-benefiting enterprises. A: *B* value in nonstandardized coefficient; B: standard error in nonstandardized coefficients; C: standardization coefficient; D: *t* value; and E: Sig.).

**Figure 12:** Test results of the mediating effect of leader narcissistic organizational identification ((a) employees' mental health and (b) employees' emotional contagion perception. A: *R*^2^; B: adjusted *R*^2^; C: *R*^2^ variable; and D: *F* value).

**Figure 13:** Analysis of the accuracy of employees' emotion ((a) training average accuracy curve, (b) verification of the average accuracy curve, and (c) comparison results of the average error rate under regression loss combination. A: Euclidean distance classification loss+average absolute error regression loss; B: Euclidean distance classification loss+variance loss; C: improved focus loss+average absolute error regression loss; D: improved focus loss+variance loss; E: cross-entropy loss+variance loss; F: cross-entropy loss+average absolute error regression loss).

**Table 1:** Statistical results of the correlation coefficients of the variables.

Variable	1	2	3	4	5	6	7	8	9	
A	1									
B	0.783^∗∗^	1								
C	0.809^∗∗^	0.429^∗∗^	1							
D	0.734^∗∗^	0.476^∗∗^	0.527^∗∗^	1						
E	0.632^∗∗^	0.406^∗∗^	0.351^∗∗^	0.284^∗∗^	1					
F	0.442^∗∗^	0.368^∗∗^	0.375^∗∗^	0.587^∗∗^	0.532^∗∗^	1				
G	0.571^∗∗^	0.301^∗^	0.231^∗∗^	0.224^∗∗^	0.641^∗∗^	0.681^∗∗^	1			
H	0.534^∗∗^	0.395^∗∗^	0.359^∗∗^	0.364^∗∗^	0.439^∗∗^	0.285^∗∗^	0.543^∗∗^	1		
I	0.538^∗∗^	0.561^∗∗^	0.274^∗∗^	0.552^∗∗^	0.368^∗∗^	0.362^∗∗^	0.567^∗∗^	0.439^∗∗^	1	
J	-0.261^∗∗^	-0.664^∗∗^	-0.271^∗∗^	-0.523^∗∗^	-0.376^∗∗^	-0.442^∗∗^	-0.551^∗∗^	-0.328^∗∗^	-0.278^∗∗^	1

Note: ^∗^significant value 0.01 < *p* < 0.05 and ^∗∗^significant value 0.001 < *p* < 0.01. A: pretending expression; B: indifferent expression; C: contempt expression; D: sincere expression; E: organizational identification; F: happy; G: frustration; H: general; I: positive attitude towards work; J: negative attitude towards work.

## Data Availability

All data are fully available without restriction.
